# TiO_2_-DNA Nanosensor In Situ for Quick Detection of Nasal Flora in Allergic Rhinitis Patients

**DOI:** 10.1155/2022/5708326

**Published:** 2022-04-13

**Authors:** Weihua Chen, Kaiyang Zhang, Zewei Zhong

**Affiliations:** Ear-Nose-Throat Department, Longyan First Hospital Affiliated to Fujian Medical University, Longyan, Fujian 364000, China

## Abstract

**Background:**

A relevant study found that allergic rhinitis (AR) may be related to the imbalance of nasal flora. Therefore, if the nasal flora of AR patients can be detected quickly, it is of great significance to study the distribution law of nasal flora in AR patients and explore its correlation with AR.

**Objective:**

To design a new and convenient nano-DNA sensor for quick screening of nasal flora in allergic rhinitis (AR) patients, so as to provide experimental basis for the prevention and treatment of AR.

**Methods:**

We create a synthesized nanostructured DNA biosensor called Nano-TiO_2_-DNA sensor which can be combined with samples from nasal mucosa or secretion with high efficiency and detect certain flora in situ without DNA extraction or RNA sequencing. In a physical property test, firstly, we tested the permeability, solubility, and storage temperature of nano-TiO_2_, so as to provide experimental basis for the synthesis of Nano-TiO_2_-DNA sensor. Subsequently, the permeability of Nano-TiO_2_-DNA sensor in Staphylococcus aureus was further tested. In a clinical experiment, we selected 60 AR patients treated in our hospital from September 2020 to September 2021 as the AR group and 60 healthy people who underwent physical examination at the same time as the control group. The Nano-TiO_2_-DNA sensor was used to detect typical nasal flora in AR patients, and Pearson's correlation analysis was used to explore the correlation between nasal flora with serum IgE and eosinophils.

**Results:**

As for physicochemical characteristics, this sensor can permeate into certain bacteria directly and specifically. It has high affinity ability with a target, and the combination can be detected by evaluating the released fluorescence qualitatively and quantitatively. It can be stored at −20°C in ethyl alcohol stably. By this sensor, we have successfully detected *Staphylococcus aureus*, *Klebsiella pneumoniae*, and *viridans streptococci* in AR patients compared with healthy people, which will help these patients in the prevention of acute sinusitis and acute or subacute pneumonia. Furthermore, we found Proteus had the strongest positive correlation with AR while Actinomyces had the biggest negative correlation.

**Conclusion:**

The Nano-TiO_2_-DNA sensor will help an outpatient doctor more for quick screening certain nasal flora in AR patients and improve the prevention of AR-related complications.

## 1. Introduction

Allergic rhinitis is a global health disease which has a profound impact on people's social work, daily life, and school events, although leading to no serious sequelae and death [1]. The worldwide incidence of AR is about 10% in adults and 40% in children [2]. The typical characteristic of AR is hyperreactivity of nasal mucosa mediated by IgE, together with a high level of eosinophils. As there are no effective prevention and radical cure at present, many AR patients, especially children, can only avoid or just alleviate the blocked, runny, and itchy nose by avoiding allergens [3, 4].

AR is associated with many factors, such as irregular work and rest, unhealthy diet, and abused or overuse of antibiotics, which make the nasal mucosa more easily and frequently exposed to foreign microorganisms and antigens [5, 6]. It has been proved that microorganisms are regarded as a necessary part in AR occurrence [7]. The imbalance of microbial flora in nasal mucosa can affect the development of immune system and make the immune response unbalanced, which easily trigger AR to some extent [8, 9]. Some researches proved that superantigens from bacteria were able to trigger high level of IgE as these superantigens have been acting as inflammatory factors for airway hyperreaction [10, 11]. Besides, AR patients tend to have acute nasal infection like acute nasosinusitis because nasal mucosa is more susceptible to bacteria resulting from broken immune defensive activity or T cell-involved inflammatory reaction [12–14]. As a result, nasal flora detection and analysis help for AR diagnosis as well as prevention of complication.

At present, the commonly used bacterial detection methods in clinic mainly include smear detection, bacterial culture, serological detection, bacterial nucleic acid detection, and second-generation sequencing, which plays a key role in the study of nasal flora distribution in AR patients, but there are also some deficiencies. For example, bacterial culture generally takes 3 days, and special flora even takes a week, which cannot meet the needs of early diagnosis. The specificity of serological antibody detection is relatively poor, which is prone to false positive or false negative results. In addition, second-generation sequencing technology and PCR amplification can go through almost all the abnormal flora distribution in nasal mucosa in detail via its high throughput detecting process [15, 16], but it is relatively expensive and time-consuming, which not facilitate some quick screening when needed. Hence, more convenient and cheaper technology are required for quick screening nasal flora which will no doubt help a physician to get a knowledge of nasal flora distribution in AR patients as soon as possible. Here, we create a synthesized nanostructured DNA biosensor called Nano-TiO_2_-DNA sensor which can be combined with samples with high efficiency and detect certain flora in situ without DNA extraction or RNA sequencing. By this method, we can easily detect known flora by observing and quantifying the releasing fluorescence from the biosensor. So far as we know, there are few clinical studies on the specific detection of flora using nano-DNA sensors, and the emergence of this technology may bring new changes to the rapid detection of microbial flora.

## 2. Materials and Methods

### 2.1. Nano-TiO_2_ Preparation and Physicochemical Property Test

TiO_2_ nanoparticles (13463-67-7, Sigma-Aldrich, MO, USA) were prepared. As these particles were used as the vector to enhance the penetration capacity of nano-DNA, here, we first packaged the particles to test its bind ability with bacteria. Hence, we first test its binding ability with bacteria by coupling fluorescein isothiocyanate (FITC). The TiO_2_-FITC was mixed with Staphylococcus aureus (ATCC25923, Thermo Fisher Scientific, Massachusetts, USA) which was stained by MycoLightRed (AAT-B22413, AAT Bioquest, CA, USA). Second, we need an appropriate medium to carry our designed DNA sensor with maximum solubility and a stable storage temperature. So, we dissolve TiO_2_-FITC in different kinds of medium including distilled water, Phosphate-Buffered Saline (PBS), methyl alcohol, ethyl alcohol, and formic acid and test the fluorescence abortion of precipitated TiO_2_-FITC after standing for 24 h away from light. After confirming the best medium, dissolved TiO_2_-FITC was stored at different levels of temperature including −80°C, −20°C, 4°C, 37°C, 58°C, and 98°C for another 24 h, and precipitated TiO_2_-FITC was tested again via fluorescence abortion. Confocal microscopy (SP8, Leica, Wetzlar, Germany) was applied for fluorescence image observation, and SpectraMax (i3X, Molecular Devices, CA, USA) was used for fluorescence quantitative analysis.

### 2.2. Nano-TiO_2_-DNA Sensor Construction

First, nanostructured DNA was designed the following steps: (1) Two separate Staphylococcus aureus-related oligonucleotides were designed. (2) FITC-labeled beacon was merged in the oligonucleotides via stirring at 60°C for 30 min and cooling down at 4°C for 5 min. (3) An fluorescence negative stop beacon tag was assembled in the opposite side of oligonucleotides after incubating at 37°C for 2 h and 60°C for 5 min with a mixture of glycerol to form the key part of the oligonucleotides which will bind to the target sequence of candidate bacteria into a ring structure, which will stop the fluorescence release. Then, TiO_2_ particles were conjugated with nano-DNA after stirring the mixture at 37°C for 12 h in borate buffer and removing free nano-DNA via centrifugation at 3000 rpm for 5 min. Dioleoyl-trimethy-lammonium-propane (DOTMA,132172-61-3, Sigma-Aldrich) was coated surrounding the TiO_2_-DNA to enhance the biocompatibility in samples with less immunological rejection, using distilled water to wash the sensor three times and store at 4°C for later use (Figure 1). Other flora-related sensors will be constructed following the above protocol when necessary.

### 2.3. Nano-TiO_2_-DNA Sensor Permeation Test

Pure nano-DNA sensor and nano-TiO_2_-DNA sensor were separately mixed with Staphylococcus aureus to compare the infiltration ability. The reaction process was 95°C for 1 min, 62°C for 3 min, and 72°C for 5 min. Thus, the fluorescence intensity was detected 10 min later by fluorescence microscopy (BX51, Olympus, Tokyo, Japan). As this sensor was designed for quick observation, no more waiting minute was needed. Besides, the fluorescence intensity detection was performed every 12 h and lasted for 72 h to test the fluorescence stability.

### 2.4. Clinical AR Patient Inclusion and Conventional Nasal Flora Detection

60 AR patients as well as the same number of healthy people who performed healthy examination in our hospital were included, all aging from 5 to 65 years. For AR patients, serum IgE and eosinophil percentage from blood were evaluated and relative data were collected from a clinical lab. All patients participating in this study voluntarily signed informed consent, and the study was approved by the medical ethics association of our college. As we plan to create a quick method to confirm the common or typical nasal flora in AR patient, here, we need to perform a conventional nasal flora examination to confirm these typical floras. Hence, nasal secretion was collected from AR patients and control people. After total DNA extraction (MagMAX-96™ DNA Multi sample kit, 4413021, Thermo Fisher Scientific, USA), 16 s rRNA primers in V1 and V2 region including 27F and 338R were used for PCR amplification. 250 bp × 2 double-terminal sequencing of PCR products was performed using the Hiseq second-generation high-throughput sequencing platform (Illumina).

### 2.5. Nano-TiO_2_-DNA Sensor Detection in Typical Nasal Flora in AR Patients

After confirming the typical nasal flora in AR patients, we selected the top three kinds of flora in AR patients and healthy people separately as a target for testing. Before performing the test, the specific sensors related to certain floras will be synthesized based on the same protocol above and then mixed with the samples which come from nasal secretion of AR patients and healthy people quickly. The results can be evaluated after 10 min, and whether the positive result matched the conventional nasal flora date would be known.

### 2.6. Correlation Analysis of Nasal Flora with IgE and Eosinophils

To support the testing result by DNA sensor and to provide some helpful information for AR prediction, we further analyzed the correlation of nasal flora with IgE and eosinophils, in order to obtain the most relevant flora with AR.

### 2.7. Statistical Analysis

SPSS 22.0 and MedCalc software were adopted for statistical analysis. The quantitative data were described by *n* (%), and the quantitative data was described by *x* ± *s*. A *t*-test was employed for intergroup comparison. Pearson's correlation analysis was used to detect the correlation between nasal flora with IgE and eosinophils. *P* < 0.05 stands for striking difference.

## 3. Results

### 3.1. Permeation Test and Physicochemical Characteristics of TiO_2_

As we selected TiO_2_ as the vector to enhance the infiltration ability of our sensor, here, we test its infiltration characteristics in flora. Obviously, TiO_2_ could permeate into Staphylococcus aureus directly (Figures 2(a)–2(i)) and presented a good colocalization with staphylococcus aureus under a confocal image. Besides, we test the solubility of TiO_2_ in some candidate media and find ethyl alcohol as the best medium to dissolve TiO_2_, with the least sediment after the solution standing by for 24 h (Figure 2(j)). Besides, the TiO_2_ had the best stable status when being stored at both −80°C and−20°C, so the constructed sensor could be stored at −20°C to maintain its stability (Figures 2(k)–2(n)).

### 3.2. Permeation Capacity Comparison of Nano-DNA Sensor and Nano-TiO_2_-DNA Sensor

Although we can synthesize the pure nanostructured DNA, it was not able to permeate the flora with high efficiency; thus, we packaged the TiO_2_ and DOTMA outside of the DNA sensor to form a Nano-TiO_2_-DNA sensor, based on the better permeation capacity of TiO_2_ and good biocompatibility of DOTMA. It was proved that the TiO_2_-DNA sensor had better permeation capacity than the pure DNA sensor (Figures 3(a)–3(f)), and it could stay inside of the target flora for as long as 60 h (Figure 3(g)).

### 3.3. Clinical Information and Conventional Nasal Flora Analysis in AR Patients

Here, we presented the age distribution of AR patients and control people with no significant difference (Figure 4(a)) and sex ratio of AR patients (Figure 4(b)). Included AR patients presented much higher level of serum IgE (Figure 4(c)) and eosinophil ratio (Figure 4(d)). To confirm the sensitivity and specificity of our designed sensor, we first analyzed the nasal flora category of included AR patients by conventional sequencing method and find some significantly high groups of flora in AR patients, among which the top three kinds of flora were *Staphylococcus aureus*, *Klebsiella pneumoniae*, and *viridans streptococci*, while *Coagulase-negative Staphylococci*, *Corynebacterium*, and *Propionibacterium acnes* were the top three of healthy people (Figure 4(e)). Hence, we tested these floras by our designed sensor to confirm its availability in quick screening.

### 3.4. TiO_2_-DNA Sensor in Quick Screening of Top Nasal Flora in AR Patients and Healthy People

Here, we applied our designed TiO_2_-DNA sensor which had separate sequence information for each kind of flora to quickly test the nasal mucosa sample from AR patients and healthy people. Consistent with the result by a conventional sequencing method, our sensor could detect *Coagulase-negative Staphylococci* (Figure 5(a)), *Corynebacterium* (Figure 5(b)) and *Propionibacterium acnes* (Figure 5(c)) with much higher fluorescence but very few number of Staphylococcus aureus (Figure 5(d)), *Klebsiella pneumoniae* (Figure 5(e)), and *viridans streptococci* (Figure 5(f)) in healthy people while the AR patients presented the totally opposite result (Figures 5(g)–5(l)). Hence, our sensor was able to be used for quick screening of nasal flora in AR patients with higher sensitivity and efficiency.

### 3.5. Correlation Analysis of Nasal Flora with IgE and Eosinophils

Next, we analyzed the correlation of the above nasal flora with the level of IgE and eosinophils, aiming to find some cues for better prevention and therapy of AR. Finally, we found that Proteus had the strongest positive correlation with AR while Actinomyces had the biggest negative correlation, as shown in Table 1 and Figure 6.

## 4. Discussion

In this study, we focus on the nasal flora in AR patients as this evidence will contribute to AR diagnosis and complication prevention caused by AR [17–19]. To quick screen the nasal flora in nasal mucosa, which will provide more convenience for outpatient physician, we develop a new method, which is nasal mucosa flora in situ detection by the Nano-TiO_2_-DNA sensor. The working principle of this kind of synthesis nanostructured DNA is the “open and shut” process for fluorescence beacon. In a pretest situation, the fluorescence beacon was silenced by a stop beacon after forming a circle structure in the DNA sequence. This silent structure has no fluorescence release, so we cannot detect any signal before mixing the sensor with samples. During the testing process, the biosensors will be mixed with samples and find their complementary sequence if they exist under a certain reaction condition. In this process, the ring structure will be opened and the silent fluorescence will be released again. Hence, if there exists a certain kind of flora in the nasal sample, we can detect the fluorescence signal, and the fluorescence intensity will reflect the quantity of certain targets. As a result, we can confirm certain flora both qualitatively and quantitatively.

This kind of sensor has the following advantage. First, this sensor is very easy for use. It can be dropped on samples which were collected from the surface of nasal mucosa directly and under a simple reaction temperature cycle without DNA extraction, PCR process, and sequencing. Thus, the sensor screening method can be realized at an outpatient department by an assistant without sending to clinical lab or even a third party of inspection company. This will save work time for a physician and save money for patients obviously. Second, the result is easy to get. As the read out is the fluorescence signal, so it is easy for judgment without too many false positive or false negative results.

By this sensor, we successfully detect some high level of flora in AR patients including Staphylococcus aureus, Klebsiella pneumoniae, and viridans streptococci. Yoo et al. [20] applied a nano-TiO_2_ biosensor to the detection of E. coli, which effectively improved the targeting and specificity of the E. coli detection, consistent with the results of the present study. To our knowledge, the above floras detected in AR patients have much correlation with body infection including acute sinusitis and acute or subacute pneumonia, so we guess this may be an explanation why some AR patents tend to suffer from these two kinds of infectious disease [21, 22]. The correlation analysis also gave out strong evidence for the link of these floras with the diseases. Hence, by our designed biosensor, we can quickly predict occurrence of sinusitis and acute or subacute pneumonia and give suggestion to patients in time for relative prevention. However, there exist obvious shortages for the sensor application; that is, these sensors are designed based on known abnormal flora in nose, which is confirmed by conventional sequencing technology. Just as being shown in our paper, we first use the conventional second generation of sequence technology to screening the relative abnormal flora in AR patients, compared with the flora in healthy people. After having a clear recognition of the flora information, we were able to design corresponding flora based on their known primer sequence. Hence, these synthesized nanostructured DNA cannot detect unknown population, and up-down screening is not available. Its best use should be quick screening for known flora. Understanding this shortage will help us to determine when to use the method in clinic.

This study mainly discussed the sensitivity of nanosensor to the detection of typical nasal flora, but the sample size is relatively small, and the pathogenesis of AR caused by flora is not studied, which should be improved in the follow-up study.

## 5. Conclusion

In this study, we developed a synthesized nanostructured DNA called TiO_2_-DNA sensor. This sensor was able to detect certain nasal flora in situ quickly without DNA extraction, PCR process, and conventional sequencing technology. We have successfully used this kind of sensor to detect *Staphylococcus aureus*, *Klebsiella pneumoniae*, and *viridans streptococci* in AR patients which will help these patients in the prevention of acute sinusitis and acute or subacute pneumonia. This method will help an outpatient doctor more for quick screening certain nasal flora in AR patients and improve prevention of AR-related complications.

## Figures and Tables

**Figure 1:** Synthesis principle and workflow of Nano-TiO_2_-DNA. (a) Working principle of Nano-TiO_2_-DNA. The silenced fluorescence beacon in the primary sensor will be open after meeting with its complementary sequence and release fluorescence which can be detected. (b) The constructing principle of Nano-TiO_2_-DNA. TiO_2_ particle-conjugated nano-DNA will be coated with Dioleoyl-trimethy-lammonium-propane. (c) Method for Nano-TiO_2_-DNA application. The sensor will be incubated with samples in situ directly for target sequence detection.

**Figure 2:** Permeation test and physicochemical characteristics of TiO_2_. (a–c) Confocal image of TiO_2_-FITC in staphylococcus aureus, ×20. (d–f) Confocal image of TiO_2_-FITC permeated staphylococcus aureus, ×20. (g–i) Confocal image of merged TiO_2_-FITC and permeated staphylococcus aureus, ×20. (j) Dissolving capacity test of TiO_2_. (k–m) Confocal image of precipitate TiO_2_-FITC after TiO_2_-FITC solution was standing by for 24 h, ×20. (n) Quantitative precipitate TiO_2_-FITC after TiO_2_-FITC solution was put on standby for 24 h.

**Figure 3:** Permeation capacity Comparison of nano-DNA sensor and Nano-TiO_2_-DNA sensor. (a–c) Permeation capacity of pure DNA sensor in Staphylococcus aureus, ×20. DNA-S: DNA sensor. (d–f) Permeation capacity of TiO_2_ DNA sensor in Staphylococcus aureus, ×20. TiO_2_-DNA-S: TiO_2_ DNA sensor. (g) Fluorescence intensity alteration of DNA sensor and TiO_2_-DNA sensor after being mixed with Staphylococcus aureus for 72 h.

**Figure 4:** Clinical information and conventional nasal flora analysis in AR patients. (a) Age distribution of AR patients and healthy people. (b) Sex ratio of AR patients. (c) Serum IgE level of AR patients and healthy people. (d) Eosinophil ratio of AR patients and healthy people. (e) Conventional sequencing analysis for nasal flora in included AR patients. ^∗∗∗^*P* < 0.001.

**Figure 5:** TiO_2_-DNA sensor in quick screening of top nasal flora in AR patients and healthy people. (a–f) TiO_2_-DNA sensor in healthy people. (g–l) TiO_2_-DNA sensor in AR patients, ×20. CNS: Coagulase-negative Staphylococci; PAC: Propionibacterium acnes; SA: Staphylococcus aureus; KP: Klebsiella pneumoniae; VS: viridans streptococci.

**Figure 6:** Correlation analysis of nasal flora with IgE and eosinophils. Red: positive correlation coefficient. Blue: negative correlation coefficient.

**Table 1:** Correlation analysis of nasal flora with IgE and eosinophils.

Item	Statistics	Coagulase-negative Staphylococci	Corynebacterium	Propionibacterium acnes	Aerococcus	Propionibacterium	Actinomyces	Staphylococcus aureus	Klebsiella pneumoniae	Viridans streptococci	Diphtheroids	Haemophilus	Proteus
IgE	*r*	-0.11	-0.21	-0.45	-0.66	-0.34	-0.74	0.56	0.49	0.47	0.66	0.65	0.72
	*P*	0.112	0.089	0.213	0.044	0.088	0.031	0.332	0.223	0.312	0.041	0.044	0.032

Eos	*r*	-0.18	-0.35	-0.42	-0.52	-0.61	-0.89	0.33	0.35	0.45	0.68	0.47	0.81
	*P*	0.109	0.298	0.065	0.051	0.044	0.021	0.223	0.142	0.056	0.045	0.067	0.022

## Data Availability

The simulation experiment data used to support the findings of this study are available from the corresponding author upon request.
